# A Bio Polymeric Adhesive Produced by Photo Cross-Linkable Technique

**DOI:** 10.3390/polym8080292

**Published:** 2016-08-10

**Authors:** Soliman Abdalla, Nabil Al-Aama, Maryam A. Al-Ghamdi

**Affiliations:** 1 Department of Medical Physics, Faculty of Science, King Abdulaziz University Jeddah, P.O. Box 80203, Jeddah 21589, Saudi Arabia; 2 Internal Medicine and Cardiology, King Abdulaziz University Medical School, Present Director of CCU & Consultant Adult Interventional Cardiologist, Jeddah 21589, Saudi Arabia; drnabilalama@yahoo.com; 3 Department of Biochemistry, Faculty of Science, King Abdulaziz University Jeddah, P.O. Box 80203, Jeddah 21589, Saudi Arabia; maaalghamdi3@kau.edu.sa; 4 Vitamin D Pharmacogenomics Research Group, King Abdulaziz University Jeddah, P.O. Box 80203, Jeddah 21589, Saudi Arabia

**Keywords:** bio-adhesives, photo cross-linkable, polycarprolacton, 2-isocyanatoethyl methacrylate, isocyanate functional-groups, degree of cross linking

## Abstract

The advantages of photo polymerization methods compared to thermal techniques are: rapid cure reactions, low energy demands, solvent free requirements and room temperature use. In order to form a macromer, polycaprolactone (PCL) was cross-linked via ultraviolet power with 2-isocyanatoethyl methacrylate. Different methods of characterization were carried out: estimation of swelling capacity, adhesive capacity (using aminated substrates), surface energy (by contact angle), and attenuated total reflectance Fourier transform infrared. In addition to these experiments, we carried out dynamical mechanical thermal analysis, thermogravimetry and thermorphology characterizations of PCL. Thus, it has been concluded that the prepared macromer could be transformed into membranes that were effective as a medical adhesive. The degree of cross linking has been estimated using two different techniques: swelling of the samples and photo cross linking of the samples with different periods of irradiation at relatively high UV-power (600 mW/cm^2^).

## 1. Introduction

Three decades ago, scientists first used polymeric adhesives (PA) in order to “weld” several layers of tissues together. Since then, the development of research in this area has been ongoing and PA can now be used in different medical applications, including: power to seal air infiltrations, hemostasis, and possible ability as drug delivery agent. With PA, one can close wounds without needles or local anesthetics. Moreover, around the world, stitching is still the most popular technique to fill different injuries. However, health professionals are increasingly using skin adhesives to substitute adhesive strips, stitches and crotchets (staples) in the fields of emergency medicine, shock, pediatrics, plastic surgeries and other surgeries. As a technique to fill different injuries, topical skin adhesives guarantee speed, reduced trauma and less pain. This is why they can be done without anesthesia and the problem of stitch removal is also eliminated. Bio-adhesives also have the leverage of bringing about excellent cosmetic results. In addition, they can be used as delivery frameworks that would be further engineered for delayed, localized release of medications, such as pain treatment drugs, antibiotics or chemotherapy. We can use them as mediums for growth factors [1,2,3,4,5] and actual cell lines for healing in tissues such as cartilage that heals poorly [6,7]. Clinical requirements must be obeyed by surgical adhesives. Two sides of the tissue must be held together for as long as necessary before being reduced to suitable bio-products [8]. In addition, an adhesive would make it possible to administer effective treatment in any environment. Fibrin-based adhesives are now the most commonly used in the medical community [9,10] along with cyanoacrylates [11,12]. Several problems are presented by the fibrin based adhesives, e.g., immunogenicity and risk of blood transmission diseases, including human immunodeficiency virus and bovine spongiform encephalopathy. On the other hand, to produce formaldehyde, there have been reports of cyano-acrylates degrading in hydrous environment, which might result in cancer or at least sores. Nowadays, other options are becoming available, with urethane-based adhesives becoming quite promising for this application, among the synthetic materials. However, even though other authors have conducted a number of studies [13,14], furthering our bid to expand the work (including pre-polymers, in particular concerning urethane applicable as bio-adhesives), these have only shown that, despite the better adhesion results, the time required for effective treatment is too long for surgical demands. More major advantages are offered by UV curable adhesives than pre-polymers systems like fast-curing rate, control of the polymerization heat evolution, and suitability for application to weakened, diseased or otherwise compromised tissue [15]. Ultraviolet (UV) irradiation curable bio-adhesives based on *N*-vinylpyrrolidone have been prepared by different authors [16]. Even though suitable adhesive strengths were presented by these adhesives, the setting time induced by UV was approximately 3 min, a value that should be improved for application in surgery. This work examines and reports on the formation of urethanes, starting with polycapro-lactone (PCL). PCL is made up of aliphatic polyester which is bio-degenerated, and has a semi-crystalline linear nature. The degeneration PCL is attributed to its sensitivity and weakness of its non-aromatic ester correlated with water-molecules in addition to the substance [10,11]. Health professionals have used this polymer in several medical applications and the US Food and Drug Administration has already approved it [12,13]. PCL is currently applied in the development of drug delivery systems [14], and resorbable stitches [15] and as a material for tissue regeneration [16,17]. In the present study, we adjusted polycaprolactone-diol with 2-isocyanatoethylmethacrylate to compose a macromer that can be strongly and easily connected using ultraviolet rays. We used Irgacure2959 as the photo initiator because it has been shown to fit well in several types of cells at different material concentrations [18,19].

## 2. Materials and Methods

### 2.1. Samples

We acquired diethyl ether, PCL with hydroxyl-end functionalized diol, and 2-isocyanatoethyl methacrylate (IEMA) from Sigma-Aldrich (Darmstadt, Germany) and Merck (Darmstadt, Germany). We acquired human plasma in the fresh frozen state from the KAU-University Hospital. Their frozen state was maintained until we were ready to put them to use. Then, in polypropylene tubes, we collected venous blood (from rabbit) with a 9:1 blood acid citrate dextrose (ACD) solution ratio and made use of them as soon as we collected them. We denoted these samples of blood ACD-RB. In addition, we have used the differential scanning calorimerty (DSC) technique (DSC822-Mettler ToledoInc, Coslada, Spain) in order to obtain a sufficiently good estimation of the cross linking degree for samples subjected to different UV irradiation doses. 

### 2.2. Preparation of Samples

Using IEMA and diethyl ether as solvent, we modified hydroxyl end functionalized PCL diol to synthesize PCL macromeres containing urethane groups. The ratio of isocyanate group (NCO) to hydroxyl groups used was 2:1. The choice of diethyl ether as solvent was for its relatively high volatility. 

Taking into account the refluxing of solvent-material and using N_2_ as general environmental ambience (without atmospheric air), we performed the reaction by stirring the two materials in a typical special glass-flask. Then, we put the flask in a 40 °C water bath.

The formation of urethane groups has been attained using the attenuated total reflection infrared spectroscopy Magma-IR spectrometer 750 from Nicolet Instrument (Champaign, IL, USA) Corp., equipped with a Golden Gate Single Reflection Diamond ATR (ATR-FTIR, Champaign, IL, USA) technique. After 24 h of biochemical reaction, all of the isocyanates’ functional groups with the formula NCO had completely reacted with the PCL hydroxyl groups. Using this scientific Spectrometer, we recorded spectra on an average of 128 samples with the excellent resolution of about 4 cm.

### 2.3. Ultra Violet Irradiation for Cross-Linked Systems Formation

Polymers can be characterized by either their degree of polymerization or their degree of cross-linking. The degree of polymerization is the number of repeat units in an average polymer chain which is the total number of repeating groups, while the degree of cross-linking means the number of groups that interconnect two materials. The degree of cross-linking is generally expressed in mole percent. The degree of cross-linking in PCL gel is very sensitive to different factors, the most important being the molecular motion of water molecules in the gel which can be obtained by measuring relaxation times and self-diffusion coefficients of water. In addition, different forms of energy can be used to initiate cross-link reactions, including ultraviolet exposure, mechanical pressure, heat, change in pH, or even nuclear radiation. When partially polymerized or unpolymerized, the resin is mixed together with certain compounds to stimulate a chemical reaction that forms cross-linked compounds. These materials have plastic property and they are called thermosetting materials. Generally, these reactions are irreversible and cause thermosetting properties.

In any hydrophilic polymer reaction, H_2_O plays the main role of plasticizer to form the suitable polymer network system. Here, free energy of mixing (DG free) from the polymer and solvent interaction can adequately assess the swelling process of the hydrogel under rubbery state. At initial conditions, the free energy is much smaller than zero while the elastic energy (DG elastic) is greater than zero when it is added to the mix energy (DG mix). Thus, the solvent will penetrate though the polymer matrix as the swelling process starts until the swelling equilibrium is attained at |Δ*G*_mix_| = Δ*G*_free_ + Δ*G* elastic. At this condition, the driving force has disappeared. More quantitative study to calculate |Δ*G*_mix_| will be carried out for PCL-IEMA system in future study Using photo cross-linking with ultraviolet technique, we prepared the cross-linked networks. Then with a 0.04 molar-solution of the IEMA we added the photo-initiator to the macromer. This was happening while the glass flask was kept in the water bath at 60 °C. Keeping the mixture with continuous stirring, we waited until all Irgacure 2959 material was dissolved. We removed the resultant solution from the water bath and irradiated it using a UV lamp (Model UVGL-48, Multiband UV, from Mineral light Lamp, San Francisco, CA, USA) for 60 s. After this period of time, we obtained a membrane.

### 2.4. Capacity of H_2_O-Sorption

Under suitable environmental conditions (e.g., good vacuum conditions), we primarily dried sample compounds until they attained an unchanging mass (W) at 60 °C. We then set these three samples in a suitable vessel with a saturated solution of CuSO_4_:5H_2_O and recorded their mass several times to achieve a maximum weight (*W*_d_). The swelling ratio is estimated as [20]:

(1) $$\text{SwellingRatio}\%=\left(\frac{W_{s}-W_{d}}{W_{d}}\right)\times 100\%$$

### 2.5. Estimation of Adhesive Capacity: Effect of Substrate

To assess the adhering capacity of the macromer, we sandwiched it (as a solution) between two gelatin sheets of dimensions 1.5 cm × 3 cm with an overlap of 1 cm in which we placed the adhesive. The final dimension of the glued gelatin films was 1.5 cm × 5 cm. We used ultra violet radiation to treat them using the same conditions as previously described by different authors [21,22,23,24]. Using this technique, we succeeded to strongly attach the substrates with films. We then subjected the gelatin sheets to the pull-out test [25,26], where the pulling velocity was 20 mm/min, and we established the distance between the probes at 1 cm. We carried out the assays at room temperature. The apparatus and the software program reported the force as a function of corresponding length. Finally, when gelatin sheets fractured or their separation increased, the test ended. In addition, we performed a negative control test by carrying out the same experimental test with a gelatin sheet without any treatment (1.5 cm × 5 cm).

### 2.6. Morphology of Samples: SEM-Examination

We performed the analyses in a scanning microscope JSM–5310 from Jeol (Peabody, MA, USA). Different magnifications were used to obtain a better view of the surfaces morphology and different cross sections of the membranes. These membranes were placed on a carbon stripe, which was carefully wrapped with a thin Cu film to permit good vision of the cross-linked systems. As cross section visualization was required, we cooled the membranes in CO_2_ under high pressure. At the moment that their temperature reached, they were readily broken.

### 2.7. Dynamic Mechanical Thermal Analysis

With the aid of dynamic mechanical thermal analysis (DMTA), we analyzed thick specimens (15.20 mm × 7.4 mm × 1.10 mm), we used a DMA 2980 dynamic mechanical analyzer (TA Instruments, Inc., New Castle, DE, USA) in the constraint layer-attenuating mode, with a typical average of 2 °C·min^−1^, for several frequencies mode (1, 5 and 10 Hz) and a displacement of 0.05 mm. 

We determined the *T*_g_ from the maximum point of the curve between tan (δ) and temperature: tan δ (tan δ = *E*″/*E*′) where *E*″ and *E*′ are the imaginary and real part of complex tension, respectively, obtained from DMTA data. 

We also obtained the experimental data of differential scanning calorimetry (DSC) at a typical thermal average of 2 °C·min^−1^. One can observe also from the DMTA trace a small inflexion in the region of 50 °C. This region is believed to correspond to the melting of some crystalline zones of the PCL.

### 2.8. Plasma Degeneration

For a period of 6 weeks, we carried out bio-self-elimination studies in human plasma. After thorough vacuum-drying of membranes, their weights were reported and they were carefully put in a glass tube. Then we added 1 mL of plasma to each membrane and incubated the glass tubes at 37 °C. After removing three samples from plasma, we used vacuum-drying and careful cleaning once more. The weight variations were reported at definite terms: 2 days, 1, 2, 4 and 6 weeks. In order to see the situation clearly, one of the three samples was retained for a further scanning electron microscopy test.

### 2.9. Surface Properties

The fact that surface energy (SE) is an important parameter affecting polymers adhesion, material wettability and even biocompatibility is widely acknowledged [25]. The measurement of contact angles is deemed the most convenient technique for the determination of the surface free energy of solid samples. This method relies on the determination of the interactions between liquids with well-determined surface tensions and the solid sample of interest. Owens, Wendt, Rabel and Kaelble, maintain that one can divide the interfacial tension in two components: dispersive interactions and polar interactions [27]. Polar interactions bring about Coulomb interactions between permanent dipoles and the ones between permanent and induced dipoles. The interactions caused by time fluctuations of the charge distribution within the molecules are known as dispersive interactions. In the course of this work, we evaluated surface energies of the cross-linked polymer and a gelatin sheet by static contact angle (θ) measurements in an OCA 20 from data physics to make a comparison between them and the published data concerning skin and blood. We carried out the necessary tests on the air-facing surfaces of the samples with different solvents such as: water, formamide, ethylene glycol and propylene glycol with the sessile technique. We performed nine measurements on different points to calculate the mean static contact angle θ and its standard deviation. We determined the dispersive (γ^S^)^D^ and polar (γ^S^)^P^ components of the urethane in addition to the one of the gelatin layers in line with the Owens-Wendt-Rabel and Kaelble relationship [28]. However, before application of photo-irradiation the adhesive should be in the liquid form. So, using the Young-Laplace method, we estimated the surface tension of the liquid adhesive with the same apparatus used during surface energy estimation. By applying this technique, we carried out the experimental data by analyzing the situation of an adhesive tinny portion or (hanged-drop) in direct contact with air through time. Using Imai and Nose’s gravimetric method [29], we estimated the rate of thrombus formation on three specimens of the membrane area. Thus, we, first, used anti-coagulated ACD-RB. Then, we prepared this sample by putting 1 mL of acid citrate dextrose solution in 9 mL of pure blood. The membranes were immersed in PBS solution at the standard environmental conditions (humidity and temperature 37 °C) before performing the tests.

After 48 h of incubation, the PBS was removed and the ACD-RB was placed in contact with the surface of the polymers and with an empty Petri dish acting as a positive control. We initiated blood clotting tests by adding 0.02 mL of a 0.10 M calcium chloride solution and stopped them after 45 min by the addition of 5 mL of water. We fixed the resultant clots with 5 mL of a 36% formaldehyde solution and then dried them with tissue paper before finally weighting them.

We followed the prescriptions of the American Society for Testing and Materials (ASTM, 2000) in performing the haemolysis tests. 7 mL of PBS have been added to 3 specimens of area 21 cm^2^ in polypropylene test tubes.

After 3 incubation days, we replaced the PBS by 1 mL of ACD-RB of concentration 9 mg/mL; here, we totally took off the PBS and put on the ACD-RB instead. Then, we set positive and negative reference samples when putting an equal quantity of ACD-RB in 7 mL of PBS and H_2_O. After 30 and 60 min, we twice inverted each of the three tubes to maintain the contact between the ACD-RB and the material. After completing the incubation process, we centrifuged the samples for 30 min for IUPAC at 2000 rpm. Using a vis spectrophotometer (Jasco V-550, Columbus, OH, USA), we estimated the rate of hemoglobin released by haemolysis. This was completed using optical densities (OD) techniques. Then, we calculated the percentage of haemolysis following Ferreira et al. [21]:

(2) $$\%\text{Haemolysis}=\left(\frac{OD_{test}-OD_{negativecontrol}}{OD_{positivecontrol}-OD_{negativecontrol}}\right)\times 100$$

## 3. Results and Discussions

### 3.1. Preparation of Samples

Reaction between polycaprolactone and its hydroxyl derivatives yields a macromer with 2-isocyanatoethyl methacrylate. The creation of urethane groups is the essential feature of this reaction. In order to be sure that the carbon double bonds terminate the urethane compound, a ratio of 2:1 of NCO/OH groups was used. Illustration on Figure 1 shows the presence of bands at 3378 cm^−1^ (N–H hydrogen-bonded stretching) and at 1525 cm^−1^ (C–N stretching and N–H bending come directly from urethane group). The functional groups NCO that asses the isocyanate chemically- interact immediately with all the hydroxyl groups in PCL. This is because we did not observe the presence of the OH groups (3492 cm^−1^) in the macromer spectra. Observations of bands at 1637 and 814 cm^−1^ show that carbon double bonds in the PCL under test are confirmed. Ultra violet photo-initiator (Irgacure 2959) was used in order to cross-link the macromer as shown in the scheme of the reactions (Figure 2). Figure 3 illustrates the ATR-FTIR spectrum of the PCL-IEMA samples. The non-attendance of the carbon double bond is the principal difference shown between the ATR-FTIR carried out before and after the ultra violet irradiation. Also, we observed that this absence occurs when irradiating with a period of time after at least one minute of UV-irradiation. As illustrated in Figure 1, (a) some hydrolysis of the ester groups enhances the partial degradation of PCL which can shift the peaks to appear at 1722, 1717 and 1715 cm^−1^ respectively. (b) The bands that appear at 3378 cm^−1^ are attributed to the formation of urethane groups (stretching of NH hydrogen). Also, one can see the stretching of CN and NH bending from the urethane group. One can also note that all hydroxyl groups of PCL reacted with NCO groups (coming from isocyanate) due to the disappearance of the band at 3492 cm^−1^. Thus, when all the isocyanates groups reacted with the PCL, the corresponding bands in IEMA spectrum disappeared. The bands at 1637 and 814 cm^−1^ reveal the presence of C=O bonds in the modified PCL. The principal difference shown between the ATR-FTIR spectra carried out before and after UV-treatment was the disappearance of the C=O band in the irradiated polymer with UV. This means that the cross linking reaction was successfully finished within one minute of irradiation. We summarize this situation in Table 1.

### 3.2. Capacity of H_2_O-Sorption

Using polymers in different medical applications is useful where the swelling capacity of the polymer plays an important role in these applications. For example, if a polymer is placed in vivo, high swelling values will be obtained leading to different side effects following the compression of the vascular structures. This will lead in turn to some effects, such as inefficient cicatrisation or different types of infections. We obtained relatively low swelling ratios that rise to about 3.21%.

### 3.3. Estimation of Adhesive Capacity: Effect of Substrate

When sandwiching an adhesive between two gelatin sheets, the binding capacity could be determined with irradiation for 1 min and subjected to binding strength examination. Here, one can use a sol sample of gelatin as control.

The values of the maximum force were registered: For a control gelatin sheet, the fracture occurred at 79.0 N and for glued gelatin at 70.7 N. Figure 4 shows this behavior where the applied force is plotted as a function of the displacement. The inset in this figure shows that 200 g mass was held at one end and it was supported for at least 20 min.

This means that the urethane was effectively binding the two sheets regardless of the glued part. We observed no elongation and the maximum force fractured the control gelatin layer.

### 3.4. Morphology of Samples: SEM-Examination

One can examine the morphology of the samples with nearly no loss of image tolerance through the analysis. We obtained different magnification SEM images as shown in Figure 5A,B. As seen from Figure 5, a uniform porous structure was detected. This was confirmed when reducing the magnification power which is clearly shown in Figure 5A.

Figure 6 shows two distinct peaks. One lies in the range −53.3 up to −52.3 °C which is insensitive to temperature but it is sensitive to the frequency. This dependence can be described by the empirical equation, at 5 Hz: $\tan d={\left(0.012+1.38/60\right)}^{\frac{p/4\times \ln2\times \text{exp}\left(-4\ln2\right)\times {\left(T+52.87\right)}^{2}}{60^{2}}}$. We believe that this is due to the glass transition effect. More calculations can be carried out to estimate the relation between the viscous forces near the glass transition point and other environmental factors such as temperature, relaxation of molecules, and addition of other chemicals. In contrast, the second peak, which is present at −10.6 °C, shows no dependence with the frequency and represents the crystallization. It is possible to observe also from the DMTA trace a small inflexion in the region of 50 °C. This region is believed to correspond to the melting of some crystalline zones of the PCL.

### 3.5. Dynamic Mechanical Thermal Analysis

Useful information on the thermal and mechanical properties was obtained using DMTA technique [30]. The gelatin will be deformed if a sinusoidal mechanical load has an effect on it. At the same time, temperature is controlled with programmable software. Different authors have used the analysis in the constrain layer damping mode with sufficient accuracy [30,31,32,33]; we follow this technique with different frequencies as shown in Figure 6 and Figure 7. These figures illustrate the unmodified PCL and the cross-linked macromer, respectively. At 210.7 K (−62.3 °C) one can notice the presence of a peak which is sensitive to the applied frequency (Figure 5). This peak was attributed to *T*_g_. Another peak, on the same Figure 5 is shown at 262.4 K (−10.6 °C) but this second is insensitive for frequency and is attributed to the crystallization.

The present results are in harmony with previously published data [34,35]. In addition, a tinny inflexion was detected at 323 K (50 °C) (Figure 5) which could be attributed to the phase change of several crystalline zones of the PCL.

Figure 7 shows a net peak at 233 K (−40 °C), which is sensitive to frequency variations. Thus, this peak is attributed to the glass transition point *T*_g_. To estimate the activation energy for alpha relaxation, we used the well known Arrhenius equation:

(3) $$\ln f=-\left(\frac{\Delta H}{RT}\right)$$

Here *f* is the frequency of analysis *R* is the gas constant, Δ*H* is the activation energy and *T* temperature in Kelvin. Noting that the activation energy Δ*H* for PCL is 42 kJ·mol^−1^ which is far lower than Δ*H* for the synthesized compound which is 124.4 kJ/mol. Figure 8 illustrates the TGA behavior of the membrane produced by photo-cross-linking and the PCL-IEMA in liquid conditions. 

The reduction of weight loss (WL) of the samples without any UV-irradiation happens in two distinct levels where the former initiates at once without any delay after 303 K (30 °C) which is nearly the melting temperature of the solvent, while the second one happens nearly at 513 K (240 °C) and could correspond to volatilization. The melting temperature of the IEMA is about 484 K (211 °C) but there are no peaks at or around this point, which indicates the absence of any un-reacted isocyanate. The first WL at 303 K (30 °C) is confirmed by the presence of some transitions for the liquid polymer detected by TGA measurements of the membrane (PCL-IEMA). Also, the WL is better seen in liquid polymer compared to the membrane, which shows a second WL at about 599 K (226 °C). These evidences permit us to draw the conclusion that compounds with similar thermal stability could be prepared by using the photo irradiation technique. Nevertheless, at 787 K (514 °C), the polymer is totally degraded and the membrane does not melt until 873 K (600 °C). This gives a net conclusion of increased thermal stability. This is important because when considering our material for biological or/and medical use, it is evidently safe to be used at normal human body temperature 310 K (37 °C) and the compound is thermally stable.

### 3.6. Plasma Self-Elimination

Figure 9 shows the WL as a function of time and one can see that bio-self-elimination in human plasma follows a logarithmic behavior in this variation which means that WL happens more importantly through the first periods (days) of incubation. We found that 0.6 of the total WL was found after two days of plasma incubation. Moreover, the sample itself lost 0.104 of its initial weight after 6 weeks. This WL occurs initially due to self-elimination due to several bio-reactions without any enzymes. In fact, this is a direct result of the sensibility of the C–O–(CH_3_) bond towards addition of H_2_O molecules to substance [36,37]. Figure 10 shows SEM images taken when incubation was totally completed. This figure illustrates the membrane morphology and clarifies the increase of pore volume that resulted from the self-elimination mechanism. One can notice that a collapse has happened when comparing the two images illustrated in Figure 10. Li et al. [38] have reported similar behavior for polycaprolactonetriolmalate. They have used this degradable biomaterial as a biological graft for bone scaffold formation. The present authors present their acknowledgments to an anonymous reviewer for pointing this out.

### 3.7. Cross Linking Estimation

The degree of cross linking has been estimated using two different techniques: swelling of the samples and photo cross linking of these samples with different periods of irradiation at relatively high UV-power (600 mW/cm^2^).

We have used the differential scanning calorimerty (DSC) technique in order to get sufficient good estimation of the cross linking degree for the samples subjected to different UV irradiation doses. We have utilized a calorimeter (DSC822-Mettler Toledo Inc.) for the DSC-characterization of PCL-IEMA sample.

The degree of cross linking is an essential issue for any cross linking reaction and in this study it has been evaluated by two different methods: First by swelling the sample and, second, by DSC thermo-gram experiments to samples subjected to different exposure time of ultraviolet irradiation. We start with the classical method: Swelling the sample. The morphology and the thickness of polymer-film are highly affected by the degree of cross-linking (DCL) and its rate of reaction [39]. The DCL increases with time then come to a saturation value [39]. In the following, a technique which could, more rapidly, produce information on the DCL including the evaluation of the solvent swelling properties of the sample is presented. As it has been shown by Flory et al. some time ago [40] the analytical point of this technique is to estimate the solvent absorption into the sample. We have precisely weighed three samples (each one about two grams) and have taken the average value of the three. Let M1 be the precise weight of the sample taken with a high precision scale. The samples were cut to a portion of about one centimeter square. At room temperature (23 °C ± 1 °C), dimethyl formamide (DMF) (Sigma Aldrich, Darmstadt, Germany) was a liquid solvent adhering to the polymer's surface, removed by fine contact with filter paper followed by immediate weighing of the swelling sample. This sample was reweighted (M2) with gain due to integration of solvent molecules with the polymer mold. The average of the three values was taken and the net weight gain ΔW is calculated as:

(4) $$\Delta W=\left(\frac{M_{2}}{M_{1}}-1\right)\times 100\%,M_{2}\geq M_{1}$$

Δ*W* is estimated as a function of time for about a quarter of an hour. Figure 11 shows the weight gain of polymer as a function of time.

Then, second we have used the differential scanning calorimerty (DSC) technique in order to get sufficient good estimation of the cross linking degree for the samples subjected to different UV irradiation doses. We have utilized a calorimeter (DSC822-Mettler Toledo Inc.) for the DSC-characterization of the PCL-IEMA sample. First, we calibrated the temperature with the extrapolated onset transition of the phase transition of a standard material (Pure indium), where all measurements have been carried out under N_2_-flow rate about 0.8 mL·s^−1^ to minimize the potential oxidative degradation. The samples (~0.01 g) were put in an Al-pan. The heating rate of the two separate pans (sample-polymer and standard material) is about 10 °C per minute and UV-power is 600 mW/cm^2^. Figure 12 shows thermograms of PCL-IEMA subjected to different time-doses (τ_ir_) of ultraviolet radiation. These doses were taken as τ_ir_ = 0, 15, 30, 45, 60, 75, and 90 s, respectively. One can notice the presence of two main features of the curves: endothermic and exothermic. Common to all investigated time doses is a melting range between 51 and 65 °C, visible as a negative peak in the endothermic thermo-grams (Figure 12).

The variation of melting point (MP) increases nearly linearly with the irradiation time dose up to about one minute. Then, it decreases with temperature. Figure 13 shows the variation of Mp with the irradiation time where it attains a maximum value at 58 seconds. The decrease of Mp with exposure time is attributed to the potential degradation of polymer with relatively high UV irradiation power (600 mW/cm^2^). However, lower UV-power lead to weaker maxima which lead to difficulties when calculating the cross linking degree of the polymer. The second relevant characteristic, the exothermic feature, is attributed to the cross linking reaction, which occurs in the temperature range 140 °C < *T* < 200 °C. Several distinct peaks are illustrated in this temperature range. These peaks are attributed to the reaction heat generated in the radical cross linking reaction. The maximum temperature corresponding to each peak *T*_max_ is varies with the irradiation time dose τ_ir_ where it passes by a maximum at an irradiation dose of 58 s. The degree of cross linking is calculated as follows. We subtracted the heat flow (*H*_0_) corresponding to reference value of un- irradiate sample from the heat flow at each maximum (*H*_max_). The degree of cross linking, *X*_c_ in PCL-IEMA sample can be estimated as:

(5) $$X_{c}=\frac{H_{\max}-H_{0}}{H_{0}}\times 100\%$$

where Figure 13 illustrates the degree of cross linking as a function of the irradiation time.

### 3.8. Surface Properties

The surface energy γ^S^ of an adhesive is an essential parameter to determine the quality of its function. γ^S^ should be less than or at least equal to the surface energy of an adherent, which is a necessary condition to fulfill good adhesion [8,40,41,42]. The present work aims essentially to estimate how well the adhesive would spread all over a bleeding surface (if possible) and in particular over the human leather or over the base of gelatin. For skin, the threshold values of γ^S^ lies in the range 38 m·Nm^−1^ < ΔES < 56 m·Nm^−1^ depending on skin-humidity and temperature [43]; while the surface tension of blood is about 55.89 m·Nm^−1^ [44]. In addition, the surface tension of the PLC-IEAM was found to be 33.51 m·Nm^−1^. γ^S^ of gelatin was found about 44.24 m·Nm^−1^ with a dispersive component (γ^S^)^D^ 5.0 m·Nm^−1^ and polar component (γ^S^)^P^ 39.24 m·Nm^−1^. For cross-linked polymer: γ^S^ 40.77 m·Nm^−1^ (γ^S^)^D^ 6.76 m·Nm^−1^ and (γ^S^)^P^ 34.01 m·Nm^−1^. One can notice that γ^S^ for gelatin, skin and blood are stronger than the surface tension of the adhesive. Consequently, the adhesive forces will be stronger than the intermolecular forces which will facilitate the spreading of the liquid adhesive. 

Using gravimetric techniques, we have estimated the rate of production of thrombus on the surface of the obtained layer. The experimental data show that, for the membrane surface test, the rate was 0.03 and it rises up to 0.038 for the blood clots. This means that the cured adhesive has thermbogenic behavior. We did not find an important difference between the two types of thrombus: One formed over control glass and the other formed over the film itself. In fact, this is due to the surface energy of urethanes because proteins are adsorbed immediately and irreversibly at the surface of the materials with high surface energy [45,46].

If one considers that coagulation is formed from consecutive steps; the first one will be the protein adhesion followed by the thrombus formation [47] where the films have thrombogenic behavior. This is of some medical importance because adhesives can be applied in bleeding situations and this material would be developed in order not only to initiate coagulation but also to stop bleeding.

Figure 14 shows: the values of the haemolysis index of the samples which are in direct contact and did not undergo any chemical-extractions, the samples that were in direct contact and incubated in PBS, and the PBS. Under different conditions, the haemolytic index was estimated from contact between the films and Acid-citrate-dextrose blood. The rates of haemolysis for several samples distributed according to the American Society for Testing and Materials Standards C756-00 ASTM 2000 is as follows: Non-haemolytic with haemolysis rate from 0 up to 2; slightly haemolytic with haemolysis rate from 2 up to 5 and haemolytic with haemolysis rate more than 5. Standard Practices for Assessment of Haemolytic Properties of Materials (USA). Light haemolytic occurs when direct contact takes place. However, the values of haemolysis decrease when extraction with PBS was carried out. These low values are caused by products which were rinsed by PBS and not by the urethane. Although there is no standard universal level of acceptable (or non-acceptable) values of haemolysis, precise estimation of tiny amounts of plasma haemoglobin could be estimated by a haemolysis test which can provide a significant screening test. One should take care when using several medical devices that would lead to haemolysis and to make sure that what we will take as medical interest is greater than the potential risks, including checking that the rates of haemolysis lie in the safe range.

## 4. Conclusions

By adjusting a hydroxyl-end functionalized PCL diol with isocyanatoethyl methacrylate, we have prepared a macromer with urethane as the effective group in PLC. The prepared macromer is transformed into membranes which were effective as an adhesive. Homogeneous morphology Experimental data with DMTA and ATR-FTIR have confirmed the creation of material through the given reaction. The obtained macromers have suffered ultra violet irradiations which lead to formation of membranes. The obtained adhesive was effective with homogeneous morphology. The weight loss in the samples that correlated with bioself-elimination reached about 10% after 6 weeks. Indirect contact and extraction with PBS solution eliminated the haemolysis within acceptable and safe ranges.

## Figures and Tables

**Figure 1:** Before ultraviolet irradiation, the spectrum of attenuated total reflectance Fourier transform infrared spectroscopy due to poly carprolacton (PCL) adjusted with 2-isocyanatoethyl methacrylate in liquid phase.

**Figure 2:** Sequences of the different reactions which lead to the formation of the thin film: (**A**) Mixture of 2-isocyanatoethyl methacrylate (IEMA) and polycaprolactone (PCL); (**B**) The mixture IEMA and PCL after ultraviolet radiation.

**Figure 3:** After ultraviolet irradiation, attenuated total reflectance Fourier transform infrared spectroscopy due to the cross linked polycarprolacton (PCL) with 2-isocyanatoethyl methacrylate in liquid phase.

**Figure 4:** The applied force as a function of displacement at ambient temperature and pressure.

**Figure 5:** Two different magnifications of the formed-membrane illustrated by scanning electron microscope: (**A**) magnification 750×; and (**B**) magnification 3500×.

**Figure 6:** Measurement of the glass transition temperature using dynamic mechanical thermal analysis (DMTA) for poly carprolacton (PCL). Tangent delta is illustrated as a function of temperature in °C. Measurements were taken at 1, 5, 10 Hz.

**Figure 7:** Measurement of the glass transition temperature using dynamic mechanical thermal analysis (DMTA) for cross linked polycarprolacton (PCL) with 2-isocyanatoethyl methacrylate macrmer. Tangent delta is illustrated as a function of temperature in °C. Measurements were taken at 1, 5, 10 Hz.

**Figure 8:** The percentage of weight loss of cross linked polycarprolacton (PCL) with 2-isocyanatoethyl methacrylate macrmer as a function of temperature in °C. Red dots represent data after ultraviolet irradiation and black squares represent data before ultraviolet irradiation.

**Figure 9:** Biodegradation of cross linked polycaprolactone (PCL) with 2-isocyanatoethyl methacrylate macrmer within a period of incubation 6 weeks. Data are shown as mean ± SME (*n* = 3).

**Figure 10:** Two different magnifications of the cross-linked samples illustrated by scanning electron microscope: (**A**) before 6 weeks incubation; and (**B**) after 6 weeks incubation.

**Figure 11:** The weight gain as a function of time.

**Figure 12:** Differential scanning calorimetric thermo-grams show the heat flow passing through PCL-2-isocyanatoethyl methacrylate (IEMA) samples as a function of temperature for different irradiation UV-doses.

**Figure 13:** Black-thick curve represents the cross linking degree through PCL-IEMA samples as a function of irradiation UV-doses in seconds. Red-thin curve shows the variation of melting point as a function of irradiation UV-doses in seconds.

**Figure 14:** Haemolytic index (HI) of the specimens with direct contact (not subjected to extraction); values HI of the specimens incubated in PBS and of the PBS extraction solution (indirect contact). Data are shown as mean ± SME (*n* = 3).

**Table 1:** This table describes the attenuated total reflection infrared spectroscopy (ATR-FTIR) spectra and its corresponding bonds: their values and where they come from.

Band, cm^−1^	Bond	Coming from
3,378 cm^−1^	N–H hydrogen bond stretching	Isocyanates group
1,525 cm^−1^	C–N stretching and N–H bending	Urethane group
3,492 cm^−1^	NCO groups	Isocyanates group
1,637 cm^−1^	carbon double bonds	modified PCL
814 cm^−1^	carbon double bonds	modified PCL
1,722 cm^−1^	carbonyl absorption in	crystalline PCL
1,455 cm^−1^	associated with the gauche isomer	The methylene groups in the amorphous regions
1,600–900cm^-1^	chain conformation	vibration of the methylene and ester groups
